# Design of Additively Manufactured Structures for Biomedical Applications: A Review of the Additive Manufacturing Processes Applied to the Biomedical Sector

**DOI:** 10.1155/2019/9748212

**Published:** 2019-03-12

**Authors:** Flaviana Calignano, Manuela Galati, Luca Iuliano, Paolo Minetola

**Affiliations:** Department of Management and Production Engineering, Politecnico di Torino, Turin 10129, Italy

## Abstract

Additive manufacturing (AM) is a disruptive technology as it pushes the frontier of manufacturing towards a new design perspective, such as the ability to shape geometries that cannot be formed with any other traditional technique. AM has today shown successful applications in several fields such as the biomedical sector in which it provides a relatively fast and effective way to solve even complex medical cases. From this point of view, the purpose of this paper is to illustrate AM technologies currently used in the medical field and their benefits along with contemporary. The review highlights differences in processes, materials, and design of additive manufacturing techniques used in biomedical applications. Successful case studies are presented to emphasise the potentiality of AM processes. The presented review supports improvements in materials and design for future researches in biomedical surgeries using instruments and implants made by AM.

## 1. Introduction

Additive manufacturing (AM), also known as 3D printing, is a relatively new technology that includes a large number of processes based on the layer-by-layer strategy to fabricate components. In contrast to conventional subtractive technologies, in which the component is fabricated by removing material from a larger raw part, using AM techniques, the final shape of the part is obtained by adding material one layer at a time. This approach has revolutionised manufacturing, and AM is today recognised as a pillar of the third industrial revolution. In line with the digital era, the only information needed to create a part by AM processes is its 3D digital model. The advantage of this kind of approach is clearly demonstrated by the design freedom [1]. Therefore, even 3D complex geometries can be easily and directly transformed into an end-usable part in only one manufacturing step without using specific tools, moulds, or dies [2]. This kind of flexibility has attracted the attention of many fields especially the medical one which was the first user of AM technologies [3]. From this point of view, what makes AM even more attractive is the possibility to use reverse engineering (RE) methodologies to obtain almost directly the 3D models for the production; for instance, of customised parts which match the patient's anatomy. Medical images acquired by tools such as computer tomography (CT) [4] or magnetic resonance imaging (MRI) are in fact currently used for such scope. On the other hand, since the AM processes are well known as rapid prototyping (RP) technique, the integration between RE and RP techniques allows the production of physical, real 3D hard copy, models of any anatomical shape for use in surgical trial, and preoperative planning of surgery and/or simulation [5]. This helps the surgeon to clearly understand the clinical situation, to train, and to be more confident during the surgery with a decrease in the operation time. The medical field constitutes a large world to be exploited for AM processes because no extra cost is needed for customization, which is the most important aspect to be considered [6]. For all of these reasons, today AM technologies play a key role in several biomedical applications that can be resumed as follows:

- Equipment [7–9] for the production of surgical supports, instruments, and tools [10]
- Physical models for visualisation [8], preoperative planning [5], testing, and educational aims
- Fabrication of customised implants for several scopes such as prostheses [11] and devices
- Biostructures for scaffolds and tissue engineering

In addition, since AM uses a digital file, the creation of a knowledge sharing platform, which is another pillar of the third industrial revolution, is facilitated. From this point of view, activities have been undertaken to create online free and open-access repositories for 3D-printable models in the fields of biology and medicine, such as the NIH 3D print exchange [12].

## 2. From Medical Data to the 3D Model for AM Processes

The literature review aims to present and discuss in detail the most representative AM technologies, covering the main research areas and case studies of applications in medicine. The AM processes present numerous features that make them suitable for biomedical applications especially if specific materials, design, and procedure are considered.

Figure 1 shows the workflow for manufacturing customized medical devices through AM starting from the acquisition of the specific patient's anatomy. In the medical field, the discipline of reverse engineering for digital data capture and processing can be combined with the one of additive manufacturing for the fabrication of the customized part directly from a 3D digital model. Three main phases can be distinguished. The first phase is the one of reverse engineering and acquisition of the patient's anatomy to convert it to digital data (point cloud). The second phase is the design phase that involves computer-aided activities such as 3D modelling with a CAD tool [13] and finite element analysis for validation of the structural resistance of the designed part [14]. In this phase, another benefit of AM can be exploited by generating complex lightweight shapes such as lattices or trabecular structures. The design parts do not have to be fully dense, and load bearing lattice structures can be integrated into portions of the part volume to reduce overall material consumption and part weight in the specific case of customised implants with an advantage for the patient's comfort.

The third and final phase is the manufacturing of the customised part by means of an AM technique, including the postprocessing operations and sterilization that are necessary for the part to be compliant with the medical specifications and requirements.

## 3. AM Processes for Medical Applications

Nowadays, AM processes that are currently used for medical applications can be grouped into two categories according to the raw material: polymers and metals. Selective laser sintering, stereolithography, and material extrusion are the most common AM techniques for polymers, while laser powder bed fusion (L-PBF) and electron beam melting (EMB) are those for metals.

### 3.1. Selective Laser Sintering

Selective laser sintering (SLS) is a powder bed technology in which a laser beam selectively sinters thin layers (from about 60 to 100 *μ*m or more) of thermoplastic powder. After a layer is finished, the build table is lowered by the layer height, fresh powder is spread over the building bed, and a new layer is defined and sintered. The build chamber can be heated during the process as well as the powder bed can be preheated before local melting with the spot of the laser. A large range of thermoplastic powders is today available for SLS. In the medical sector, this technique is mostly used for the fabrication of visualisation models, surgical tools, and customised implants. A polyamide guide to position the osteotomized bony fragments during a zygomatic osteotomy has been developed by Herlin et al. [15]. Pilot models for preoperative planning and testing have been produced using nylon powders [16]. Mixes between oxide ceramics and a PEEK and PLC compound have been studied by Shishkovsky and Scherbakov [17] to produce porous tissue engineering scaffolds. Scaffolds for growing specific tissues have been also studied by several researchers [18–25]. Most of them demonstrated the efficiency to sustain cell growth by studying different structures and postprinting functionalization. Recent overviews [26, 27] resumed the current applications of this technology in tissue engineering. The potentiality of the SLS process compared to traditional milling has been showed by Probst et al. [28], while Pallari et al. [29] demonstrated the feasibility of customised orthosis for large production.

### 3.2. Stereolithography

The stereolithography (SLA) process first appeared in 1981, when the Japanese researcher Dr. Hideo Kodama of Nagoya Municipal Industrial Research Institute published his account of a functional rapid-prototyping system using photopolymers. Three years later, in 1984, Charles (Chuck) W. Hull made 3D-printing history by inventing SLA and co-founding the 3D Systems company to commercialize it. SLA is today referred to a certain number of AM technologies in which a liquid resin is converted into a solid part by exposing the material to a light source which selectively activates the polymerisation of the material. The older system utilises a vat of liquid photopolymer resin cured by an ultraviolet (UV) laser to create a solid 3D model. A UV laser beam is directed by a computer-controlled mirror onto the surface of the photopolymer resin to draw one cross-section of the CAD model of the part. After creating one layer, the building platform is lowered into the vat and then the laser beam tracing process is repeated. Generally, a blade is used to make a smooth resin layer. The process continues layer-by-layer until the fabrication of the part is completed. Once the model is complete, the platform rises out of the vat and the excess resin is drained. The model is then removed from the platform and placed in a UV oven for final curing in order to meet the required strength of the material. Subsequently, the supports are finally detached.

Another SLA system is known as inverted SLA because the object is built using an upside-down approach. In this case, the light source hits the material through the bottom of the vat. The process starts lowering the build platform to touch the bottom of the resin-filled vat and then moving upward of a quantity equal to the layer thickness. The UV laser then acts on the bottom-most layer through the transparent vat bottom. An advantage of this kind of system is that the build volume can be bigger than the vat itself. In addition, since the object is incrementally raised, the resin that is not solidified by the laser remains in the vat and can be reused for the next layer. One similar approach is adopted for the digital light processing (DLP) [30], another SLA system in which the UV laser is replaced by a digital projector [31]. The projector is a digital screen which flashes a single image of each layer across the entire platform. Since each layer will be composed of square pixels, the resolution of a DLP printer corresponds to the pixel size, whereas in the SLA system, the resolution is determined by the spot size of the laser.

Several resins have been developed over the past two decades, and the properties of SLA parts are continuously improving, making them not only useful as prototypes but also as functional parts. Photopolymers lack of stability in the long-time period. The high precision of the process, with a layer thickness that can be adjusted from 25 to 100 *μ*m, makes SLA suitable for producing accurate models.

The combination of medical imaging and SLA has been used to fabricate models or moulds for the preparation of implants in cranial surgery [29, 32], customized heart valves [33], ear-shaped implants [34], and aortas [35]. Dental applications are increasing [36] as well as the fabrication of tissue engineering scaffolds [37, 38], thanks also to the development of biodegradable macromers and resins [39].

### 3.3. Material Extrusion

Fused deposition modeling (FDM) is an AM process that belongs to the material extrusion category. This technology was developed by Scott Crump in the late eighties of last century, and it was marketed in the 90s by Stratasys company, of which Crump was the co-founder [40]. Stratasys holds this trade name for FDM even if the patent expired in 2009. For this reason, the subsequent printer manufacturers exploiting the same extrusion principle have coined the alternative acronym of FFF (fusion filament fabrication). FDM printers build parts layer-by-layer using a thermoplastic filament that is heated to a semiliquid state, extruded, and deposited on the printing bed along with a computer-controlled path [41]. The FDM filaments come in two standard sizes with a diameter of 1.75 mm or 2.85 mm. Depending on the size of the extrusion nozzle, the layer thickness can vary from about 50 to 500 *μ*m. As for all AM processes, the smaller is the thickness of the layer, the higher is the part accuracy but also the longer the manufacturing time. Thanks to the solid material that feeds the 3D printer, multiple extruders can be used to combine diverse materials with different properties (e.g., rigid and flexible) or colours in the single layer or in different layers.

Polylactic acid (PLA) and acrylonitrile butadiene styrene (ABS) are the two thermoplastic materials most commonly used in FDM. Lactic acid-based polymers, including PLA and PCL, have biocompatible and biodegradable properties, and hence are extensively used for medical and pharmaceutical applications. Polycarbonate-ISO (PC-ISO), in its raw state, is compliant with ISO 10993 and USP Class VI certifications used to establish biocompatibility. These biocompatible materials enable manufacturers of medical devices to rely on the FDM technique to produce devices that can be used safely for clinical trials and for low-volume productions of end-use parts. Polymethyl methacrylate (PMMA) filament was used for 3D-printing of porous patient-tailored implants for craniofacial reconstructions and orthopedic spacers [42]. On modified FDM printers [43, 44], the possibility to directly extrude polymeric compounds from pellet feedstocks offers the potentiality to extend the range of materials for biomedical applications. However, there is no evidence of specific case studies so far.

### 3.4. Laser Powder Bed Fusion (L-PBF)

Laser powder bed fusion (L-PBF), also known as selective laser melting (SLM), is an AM process that uses a high-energy density laser, usually an ytterbium fibre laser, to fuse selected areas on a single layer according to the processed data and create 3D metal parts layerwise. The building process begins with laying a fine metallic powder layer on a substrate plate in a controlled inert environment. After selective melting, the building platform is lowered, and a new layer is applied. The process is repeated until the part build height is reached. The layer thickness can vary from 15 to 150 *μ*m. The laser beam focus is controlled by a galvanometer, and the movement of the beam is controlled by an F-theta lens. In L-PBF, laser power, scanning speed, hatching distance, and layer thickness are the common process parameters adjusted to optimize the process. These parameters affect the volumetric energy density that is available to heat up and melt the powders, mechanical properties, and surface roughness of the parts produced [45]. The alloys currently available for this process include stainless steel, cobalt chromium (Co-Cr alloys), Ni-based alloys, aluminium (Al-Si-Mg alloys), and titanium (Ti6Al4V alloy). Compared with the cast and forged components, a part produced by the L-PBF process has excellent mechanical properties, thanks to characteristics of grain refinement, extended solid solubility, chemical homogeneity, reduction in quantity, and size of phase segregation [46]. However, due to the Marangoni convection induced by high thermal capillary forces, the melt pool may be unstable causing microstructures uncontrollability [47]. Therefore, to meet the current clinical requirements in parts of Ti6Al4V produced by L-PBF, heat treatment is needed to adapt the physiochemical properties and to homogenize the metal microstructures, trying to possibly improve the cytocompatibility in vitro.

### 3.5. Electron Beam Melting

Electron beam melting (EBM) or electron powder bed fusion (E-PBF) is an AM process for metal powders. In this case, the energy of an electron beam is used to melt the powder, after a preheating phase of the powder layer. The mechanic of an EBM system mixes the hardware of a welding machine and the operating base of an electron microscope [48]. The EBM® technology is still an exclusive of ARCAM AB [48], which recently introduced a specific line of machines for biomedical application such as the Q10 plus model in which the improved beam control allows a better definition of the spot size [49]. If compared to the previous model (A-machines), the Q-machines have a camera, Q-Cam, which takes a picture of each layer after the melting phase. With the aid of image-processing software, the machine provides a report about the final quality of the printed parts. In this way, defects or errors can be detected and recognised immediately, without the need for additional part inspection after production. The EBM systems work under vacuum to avoid the beam to be deflected by the air molecules. Due to the vacuum and the preheating step, the build chamber is warm during the process. Therefore, after the process, the parts need to be cooled down. At the end of the process, when the part is removed from the building chamber, a soft agglomerate of powder adheres to the surface of the built and covers it completely [50]. This agglomerate is removed by sandblasting in which the same powder of the EBM process is used in order to avoid powder contamination. After this phase of cleaning, the unused powder can be recycled several times without altering its chemical composition or physical properties, because no oxygen is present inside the building chamber during the melting process, thanks to the vacuum [50]. Because of the warm environment during the process, the part shows low residual stress as compared to laser-based L-PBF systems, which require the postprocessing of built parts by a stress-relieving treatment [51]. On the other hand, the L-PBF technique offers a better surface finish, thanks to a smaller beam size and smaller layer thickness when compared to the EBM technology [51]. However, the surface roughness resulting from the EBM process represents an advantage for medical applications. In general, Ti6Al4VELI and CoCr are the most frequently used material for medical implants produced by EBM. Patient-customised implants with high biocompatibility and structures with osseointegration properties have been developed and implemented [52–58]. A significant successful example is the large-scale production of titanium acetabular cups manufactured by two Italian companies, Lima Ltd, and Ala Ortho Srl.

## 4. Conclusions

The purpose of the current review is to provide a short summary that can give an overview of the AM applications in the medical field even to a reader who approaches the topic for the first time. The main features of each AM process have been presented also by highlighting its peculiarities and differences. Numerous references have been provided to show applicative case studies, demonstrating the potentiality of AM in the medical sector. A special effort was dedicated to providing case studies which reported not only the feasibility for large-volume production but also the indication of industries which already use additive technologies as the only manufacturing system to fabricate their medical products. Even if applications in the biomedical sector have been the first for layerwise technologies almost 20 years ago, this review showed that the research is currently active and aimed at improving the part design and extending the number of materials available for AM, as supported by the numerous studies.

## Figures and Tables

**Figure 1:** Flowchart from medical data to the final part.

## References

[1] Gibson I., Rosen D. W., Stucker B. (2010). *Additive Manufacturing Technologies*.

[2] Hopkinson N., Dickens P. (2006). Emerging rapid manufacturing processes. *Rapid Manufacturing: An Industrial Revolution for the Digital Age*.

[3] Giannatsis J., Dedoussis V. (2009). Additive fabrication technologies applied to medicine and health care: a review. *International Journal of Advanced Manufacturing Technology*.

[4] Vitković N., Mladenović S., Trifunović M. (2018). Software framework for the creation and application of personalized bone and plate implant geometrical models. *Journal of Healthcare Engineering*.

[5] Singare S., Lian Q., Ping Wang W. (2009). Rapid prototyping assisted surgery planning and custom implant design. *Rapid Prototyping Journal*.

[6] Zanetti E. M., Aldieri A., Terzini M. (2017). Additively manufactured custom load-bearing implantable devices: grounds for caution. *Australasian Medical Journal*.

[7] Patel S. R., Ghose K., Eskandar E. N. (2014). An open source 3-D printed modular micro-drive system for acute neurophysiology. *PLoS One*.

[8] McDougal R. A., Shepherd G. M. (2015). 3D-printer visualization of neuron models. *Frontiers in Neuroinformatics*.

[9] Baden T., Chagas A. M., Gage G. (2015). Open Labware: 3-D printing your own lab equipment. *PLoS Biology*.

[10] Salmi M., Paloheimo K.-S., Tuomi J., Wolff J., Mäkitie A. (2013). Accuracy of medical models made by additive manufacturing (rapid manufacturing). *Journal of Cranio-Maxillofacial Surgery*.

[11] Parthasarathy J., Parthiban J. Rapid prototyping in custom fabrication of titanium mesh implants for large cranial defects.

[12] NIH 3D Print Exchange (November 2018). Online repository for 3D-printable models for biology and medicine. https://3dprint.nih.gov/.

[13] Venne G., Esau G., Bicknell R. T. (2018). 3D printed anatomy-specific fixture for consistent glenoid cavity position in shoulder simulator. *Journal of Healthcare Engineering*.

[14] Salmi A., Calignano F., Galati M. (2018). An integrated design methodology for components produced by laser powder bed fusion (L-PBF) process. *Virtual and Physical Prototyping*.

[15] Herlin C., Koppe M., Béziat J.-L., Gleizal A. (2011). Rapid prototyping in craniofacial surgery: using a positioning guide after zygomatic osteotomy—a case report. *Journal of Cranio-Maxillofacial Surgery*.

[16] Berry E., Brown J. M., Connell M. (1997). Preliminary experience with medical applications of rapid prototyping by selective laser sintering. *Medical Engineering & Physics*.

[17] Shishkovsky I., Scherbakov V. (2012). Selective laser sintering of biopolymers with micro and nano ceramic additives for medicine. *Physics Procedia*.

[18] Chua C. K., Leong K. F., Tan K. H., Wiria F. E., Cheah C. M. (2004). Development of tissue scaffolds using selective laser sintering of polyvinyl alcohol/hydroxyapatite biocomposite for craniofacial and joint defects. *Journal of Materials Science: Materials in Medicine*.

[19] Tan K. H., Chua C. K., Leong K. F. (2003). Scaffold development using selective laser sintering of polyetheretherketone-hydroxyapatite biocomposite blends. *Biomaterials*.

[20] Adamzyk C., Kachel P., Hoss M. (2016). Bone tissue engineering using polyetherketoneketone scaffolds combined with autologous mesenchymal stem cells in a sheep calvarial defect model. *Journal of Cranio-Maxillofacial Surgery*.

[21] Liao H.-T., Lee M.-Y., Tsai W.-W., Wang H.-C., Lu W.-C. (2016). Osteogenesis of adipose-derived stem cells on polycaprolactone-β-tricalcium phosphate scaffold fabricated via selective laser sintering and surface coating with collagen type I. *Journal of Tissue Engineering and Regenerative Medicine*.

[22] Lohfeld S., Cahill S., Barron V. (2012). Fabrication, mechanical and in vivo performance of polycaprolactone/tricalcium phosphate composite scaffolds. *Acta Biomaterialia*.

[23] Zhou W. Y., Lee S. H., Wang M., Cheung W. L., Ip W. Y. (2008). Selective laser sintering of porous tissue engineering scaffolds from poly(l-lactide)/carbonated hydroxyapatite nanocomposite microspheres. *Journal of Materials Science: Materials in Medicine*.

[24] Simpson R. L., Wiria F. E., Amis A. A. (2008). Development of a 95/5 poly(L-lactide-co-glycolide)/hydroxylapatite and *β*-tricalcium phosphate scaffold as bone replacement material via selective laser sintering. *Journal of Biomedical Materials Research Part B: Applied Biomaterials*.

[25] Saska S., Pires L. C., Cominotte M. A. (2018). Three-dimensional printing and in vitro evaluation of poly(3-hydroxybutyrate) scaffolds functionalized with osteogenic growth peptide for tissue engineering. *Materials Science and Engineering: C*.

[26] Miar S., Shafiee A., Guda T. (2018). Additive Manufacturing for Tissue Engineering. *3D Printing and Biofabrication*.

[27] Youssef A., Hollister S. J., Dalton P. D. (2017). Additive manufacturing of polymer melts for implantable medical devices and scaffolds. *Biofabrication*.

[28] Probst F. A., Metzger M., Ehrenfeld M., Cornelius C.-P. (2016). Computer-assisted designed and manufactured procedures facilitate the lingual application of mandible reconstruction plates. *Journal of Oral and Maxillofacial Surgery*.

[29] Pallari J. H. P., Dalgarno K. W., Woodburn J. (2010). Mass customization of foot orthoses for rheumatoid arthritis using selective laser sintering. *IEEE Transactions on Biomedical Engineering*.

[30] Fantino E., Chiappone A., Roppolo I. (2016). 3D printing of conductive complex structures with in situ generation of silver nanoparticles. *Advanced Materials*.

[31] De Santis R., D’Amora U., Russo T. (2015). 3D fibre deposition and stereolithography techniques for the design of multifunctional nanocomposite magnetic scaffolds. *Journal of Materials Science: Materials in Medicine*.

[32] D’Urso P. S., Earwaker D. J. (2000). Custom cranioplasty using stereolithography and acrylic. *British Journal of Plastic Surgery*.

[33] Wurm G., Tomancok B., Holl K., Trenkler J. (2004). Prospective study on cranioplasty with individual carbon fiber reinforced polymere (CFRP) implants produced by means of stereolithography. *Surgical Neurology*.

[34] Sodian R., Loebe M., Hein A. (2002). Application of stereolithography for scaffold fabrication for tissue engineered heart valves. *ASAIO Journal*.

[35] Naumann A., Aigner J., Staudenmaier R. (2003). Clinical aspects and strategy for biomaterial engineering of an auricle based on three-dimensional stereolithography. *European Archives of Oto-Rhino-Laryngology*.

[36] Dawood A., Marti B. M., Sauret-Jackson V., Darwood A. (2015). 3D printing in dentistry. *British Dental Journal*.

[37] Wallace J., Wang M. O., Thompson P. (2014). Validating continuous digital light processing (cDLP) additive manufacturing accuracy and tissue engineering utility of a dye-initiator package. *Biofabrication*.

[38] Dean D., Wallace J., Siblani A. (2012). Continuous digital light processing (cDLP): highly accurate additive manufacturing of tissue engineered bone scaffolds. *Virtual and Physical Prototyping*.

[39] Sodian R., Fu P., Lueders C. (2005). Tissue engineering of vascular conduits: fabrication of custom-made scaffolds using rapid prototyping techniques. *Thoracic and Cardiovascular Surgeon*.

[40] Matsuda T., Mizutani M., Arnold S. C. (2000). Molecular design of photocurable liquid biodegradable copolymers. 1. Synthesis and photocuring characteristics. *Macromolecules*.

[41] Minetola P., Galati M. (2018). A challenge for enhancing the dimensional accuracy of a low-cost 3D printer by means of self-replicated parts. *Additive Manufacturing*.

[42] Espalin D., Arcaute K., Rodriguez D., Medina F., Posner M., Wicker R. (2010). Fused deposition modeling of patient-specific polymethylmethacrylate implants. *Rapid Prototyping Journal*.

[43] Volpato N., Kretschek D., Foggiatto J. (2015). Experimental analysis of an extrusion system for additive manufacturing based on polymer pellets. *International Journal of Advanced Manufacturing Technology*.

[44] Liu X., Chi B., Jiao Z., Tan J., Liu F., Yang W. (2017). A large-scale double-stage-screw 3D printer for fused deposition of plastic pellets. *Journal of Applied Polymer Science*.

[45] Calignano F., Cattano G., Manfredi D. (2018). Manufacturing of thin wall structures in AlSi10Mg alloy by laser powder bed fusion through process parameters. *Journal of Materials Processing Technology*.

[46] Trevisan F., Calignano F., Aversa A. (2018). Additive manufacturing of titanium alloys in the biomedical field: processes, properties and applications. *Journal of Applied Biomaterials & Functional Materials*.

[47] Antony K., Arivazhagan N. (2015). Studies on energy penetration and Marangoni effect during laser melting process. *Journal of Engineering Science and Technology*.

[48] Galati M., Iuliano L. (2018). A literature review of powder-based electron beam melting focusing on numerical simulations. *Additive Manufacturing*.

[49] Galati M., Snis A., Iuliano L. (2018). Experimental validation of a numerical thermal model of the EBM process for Ti6Al4V. *Computers & Mathematics with Applications*.

[50] Biamino S., Penna A., Ackelid U. (2011). Electron beam melting of Ti-48Al-2Cr-2Nb alloy: microstructure and mechanical properties investigation. *Intermetallics*.

[51] Froes F., Dutta B. (2014). The additive manufacturing (AM) of titanium alloys. *Advanced Materials Research*.

[52] Harrysson O. L. A., Cansizoglu O., Marcellin-Little D. J., Cormier D. R., West H. A. (2008). Direct metal fabrication of titanium implants with tailored materials and mechanical properties using electron beam melting technology. *Materials Science and Engineering: C*.

[53] Palmquist A., Snis A., Emanuelsson L. (2013). Long-term biocompatibility and osseointegration of electron beam melted, free-form–fabricated solid and porous titanium alloy: experimental studies in sheep. *Journal of Biomaterials Applications*.

[54] Heinl P., Rottmair A., Körner C., Singer R. F. (2007). Cellular titanium by selective electron beam melting. *Advanced Engineering Materials*.

[55] Thomsen P., Malmström J., Emanuelsson L. (2008). Electron beam-melted, free-form-fabricated titanium alloy implants: material surface characterization and early bone response in rabbits. *Journal of Biomedical Materials Research Part B: Applied Biomaterials*.

[56] Parthasarathy J., Starly B., Raman S., Christensen A. (2010). Mechanical evaluation of porous titanium (Ti6Al4V) structures with electron beam melting (EBM). *Journal of the Mechanical Behavior of Biomedical Materials*.

[57] Harrysson O., Deaton B., Bardin J. Evaluation of titanium implant components directly fabricated through electron beam melting technology.

[58] Heinl P., Müller L., Körner C., Singer R. F., Müller F. A. (2008). Cellular Ti-6Al-4V structures with interconnected macro porosity for bone implants fabricated by selective electron beam melting. *Acta Biomaterialia*.

